The article "Application of deep learning in automatic detection of technical and tactical indicators of table tennis" was retracted in 2023. Reasons: unreliable results or conclusions; concerns about the peer review.

# Application of deep learning in automatic detection of technical and tactical indicators of table tennis

**DOI:** 10.1371/journal.pone.0245259

**Published:** 2021-03-09

**Authors:** Fufeng Qiao

**Affiliations:** College of general education, Qingdao Huanghai University, Qing’ Dao, Shandong, China; University College London, UNITED KINGDOM

## Abstract

A DCNN-LSTM (Deep Convolutional Neural Network-Long Short Term Memory) model is proposed to recognize and track table tennis’s real-time trajectory in complex environments, aiming to help the audiences understand competition details and provide a reference for training enthusiasts using computers. Real-time motion features are extracted via deep reinforcement networks. DCNN tracks the recognized objects, and the LSTM algorithm predicts the ball’s trajectory. The model is tested on a self-built video dataset and existing systems and compared with other algorithms to verify its effectiveness. Finally, an overall tactical detection system is built to measure ball rotation and predict ball trajectory. Results demonstrate that in feature extraction, the Deep Deterministic Policy Gradient (DDPG) algorithm has the best performance, with a maximum accuracy rate of 89% and a minimum mean square error of 0.2475. The accuracy of target tracking effect and trajectory prediction is as high as 90%. Compared with traditional methods, the performance of the DCNN-LSTM model based on deep learning is improved by 23.17%. The implemented automatic detection system of table tennis tactical indicators can deal with the problems of table tennis tracking and rotation measurement. It can provide a theoretical foundation and practical value for related research in real-time dynamic detection of balls.

## 1. Introduction

Image extraction, data analysis, and deep learning technologies are widely applied as big data and artificial intelligence develop rapidly [1]. Among the various applications, sports and e-sports industries change more notably. The auxiliary systems of various competitions in these industries are of great significance for tactical analysis [2]. These data provide the measurement standard for teams and fans to judge athletes’ performance and help athletes find their technical defects for targeted training. Data statistics can also improve the accuracy of games and tactical predictions [3]. However, the sports industry’s tactical data are generated manually through simple algorithms before the data explosion, ineffective and fallible [4]. Therefore, improving detection algorithms is vital to technicalize the sports industry [5]. Table tennis is a competitive sport popular in China; however, this game rarely has mature statistics systems [6]. The game videos’ characteristics are the fundamental cause. First, the tiny table tennis balls move fast, which are hard to locate and track [7]. Second, unlike other sports, table tennis ball’s rotation information is vital during competitions. The video data must have clear images to calculate the ball’s rotation and a high camera frame rate to correctly judge the rotation speed. Furthermore, the camera hardware must be advanced, limiting the generation system’s development significantly [8]. Therefore, real-time monitoring and controlling prediction are urgent problems in sophisticated environments.

A mobile camera robot is common for detecting table tennis’s technical indicators [9], aiming to detect the ball’s position and predict its trajectory in momentary time. The basis of robot design is quickly obtaining accurate information [10]. Peng et al. (2016) processed data in table tennis competitions using a big data analysis algorithm. This approach could effectively analyze the technical and tactical statistical systems and data [11]. According to the actual analysis, Wu et al. (2017) proposed the iTTVis (Interactive Visualization of Table Tennis Data) system. This novel, interactive table tennis visualization system supported the detection of tactical patterns of statistical and scoring time and allowed cross analysis to obtain tactical points [12]. Hung et al. (2018) proposed a new algorithm that could automatically find the ball’s position and racket in the image captured by the high-speed camera, which provided an objective factual basis for the referee to determine by analyzing the motion trajectory [13]. Hegazy et al. (2020) proposed a FastDTW (Fast Dynamic Time Warping) method based on a deep infrared camera. This method could detect players’ hitting efficiency to enhance the training experience; besides, its detection accuracy was 88%-100%, which was improved compared with the traditional methods [14]. The above studies suggest that different hardware facilities and processing methods have been employed to improve table tennis’s tactical analysis; nevertheless, research on the algorithms is little. Therefore, problems in analyzing and detecting table tennis competitions are researched based on hardware construction.

The aim is to track and predict the trajectory of table tennis balls. On this basis, the physical model for the ball’s flight prediction is equipped with a high-speed camera. Most of the physical models are quite complicated; hence, machine learning is adopted to predict the trajectory of the table tennis ball. A ball tracking system, a feature extraction system, and a ball trajectory prediction system are included to obtain better predictions. The novelty is that the flight trajectory between the service point and the end of the robotic arm is treated as two parabolas; the DDPG algorithm is fused with deep learning; the information and laws of the feature points on the table tennis ball in multiple consecutive frames of images are utilized to estimate the speed of the ball and the information line of the rotation axis. The table tennis trajectory is predicted and analyzed in real-time through the LSTM algorithm.

## 2. Methods

### 2.1 Traditional recognition and detection algorithms of table tennis

The traditional table tennis recognition process is shown in Fig 1. The specific process is as follows: first, the image is preprocessed. The collected image is compared with the pre-collected background image to determine whether there are moving objects in those areas in the image. The image is converted from RGB to HSV space, and the filtered image is compared with the area similar to the table tennis ball in the filtered image according to the color characteristics of the ball. Then the suspected area is searched through particular contour search rules. Finally, the algorithm is designed according to the shape feature of the table tennis ball and obtains the center coordinates [15]. However, because the table tennis ball is tiny, the pixel information is insufficient so that the detectable features cannot distinguish the ball from the background of a similar color. Second, the table tennis ball moves fast; the low frame rate of the camera will blur the motion of the table tennis ball. Finally, in the rotation speed measurement, sufficient spherical information is often needed, which will cause the shooting camera to narrow the field of view and lose a lot of information [16].

**Fig 1:** A demonstration of traditional recognition and detection algorithms of table tennis.

### 2.2 Automatic detection system of table tennis tactical indicators

The automatic detection of table tennis’ tactical planning is divided into three processes. The first process is the target extraction. The proposed DDPG detection algorithm finds the ball’s area and takes it as the tracking algorithm’s display module. The foreground area is extracted by background subtraction to narrow the search range. The target’s initial position needs to be found in the first few frames and tracked through the algorithm’s other steps. Second, CNN tracks the model. If the target is found in the previous frame, it is used as the tracker. The candidate area near the current target position is the input. Before inputted into the network in one or more batches, the candidate area is expanded by several pixels to ensure that the complete target can be included. The last process is the trajectory prediction. After this sequence is input into the LSTM model, the subsequent coordinate sequence can be generated automatically. Then, the trajectory and hitting point can be predicted. The parameters of the Gaussian Mixture Model are output, which is similar to the Kalman Filter. The purpose is to predict the possible position of tracking targets in the next frame and reduce the search range of tracking. The specific process is shown in Fig 2.

**Fig 2:** Flowchart of the tactical indicator in an automatic detection system.

For the combination of algorithms, the detection module is utilized first to obtain the candidate areas for screening input. Since the motion of the target object is usually continuous, the candidate area far away from the position of the previous frame can be excluded. The context of the previous frame’s position is also used as a candidate area. Then the candidate areas are input into the CNN model, which will return the probability value and bounding box of each area. When all probability values are lower than a set threshold, the algorithm judges that this tracking fails. Otherwise, the algorithm selects the highest probability value and the corresponding bounding box. Finally, according to the magnitude of the probability value, the bounding box is returned directly, or the bounding box size and the previous frames are averaged and returned. The reason for proceeding with this step is that the size of the bounding box changes slowly in a short time, and the size of the bounding box output by the CNN model fluctuates. When the probability value is greater than a higher threshold, the framework considers the output of CNN to be more reliable. Otherwise, based on the above assumptions, the average with the previous frames is taken. In the actual measurement, when the averaging method is not used, the tracker is prone to a particular prediction that the bounding box is larger than the actual one, which causes the search box to be too large and cannot detect the target inside it, resulting in tracking failure. When a single tracking fails, the algorithm will also use the next frame coordinates predicted by the trajectory prediction model as the tracking result according to the number of consecutive failures, or determine that the entire tracking process has failed, and repeat the first step of the framework to search for tracking targets in the entire image. Usually, tracking failures only occur when the table tennis ball flies out of the field of view or far away from the camera. Since this framework only focuses on the tracking of the table tennis ball above the table, these failures do not have much impact on the work of the framework.

### 2.3 Feature extraction based on deep reinforcement leaning

Deep learning is a multi-layer neural network obtained by simulating the analysis and feature judgment of human brain neurons. With its excellent learning ability, it has made breakthroughs in the fields of image, speech, and text. According to different application fields, deep learning networks include Convolutional Neural Networks (CNNs), Recurrent Neural Networks (RNNs), Boltzmann machines, and automatic encoders.

DDPG algorithm, a deep reinforcement leaning algorithm, contains two parts. Its structure is shown in Fig 3. The first part is Policy Gradient, a reinforcement learning algorithm based on probability. Policy Gradient represents the optimal decision during Markov Decision-Making with *π*(*α*|*s*)*Q*^*π*^ [17]. Action generation is random. In each decision-making process, the algorithm needs to integrate the whole action space:

$$\Delta \theta =\int_{s}\int_{A}p(s)\pi (\alpha |s)Q^{\pi }(s,\alpha )dads$$ (1)

The second part is the critic network. Because the algorithm uses a convolutional network or fully-connected network to approximate the value function, it is also called a value function network. The input is the action *a* and the current state *s*, and the output is *Q (s*, *a)*. The parameter updating method of the value function network is similar to that of DQN (Deep Q-Network), which is conducted to make the square of estimated and actual *Q* values smaller. The estimated *Q* value can be obtained through the state estimation network. The actual *Q* value is the sum of the output *Q* value in the state reality network (the input is the next state *S*_*t+l*_, and the action output of reality network is *a*_*t+l*_) and the real-time income *R* [18].

$$y_{t}=r(s_{t},a_{t})+\gamma Q(S_{t+1},\mu (S_{t+1}|\theta^{Q}))$$ (2)

$$\min Loss=\min\frac{1}{N}{\sum_{i=1}^{N}\left(yi-Q(S_{i},a_{i}|\theta^{Q})\right)}^{2}$$ (3)

In (2) and (3), *θ*^*Q*^ is the weight parameter of the critic network, *s*_*t*_ is the input state at time *t*, *a*_*t*_ is the output action in the input state at time *t*, *r*(*s*_*t*_,*a*_*t*_) is the immediate benefit of the action *a*_*t*_ at *s*_*t*_, *Q*(*S*_*i*_,*a*_*i*_|*θ*^*Q*^) represents the output of the critic network, and *μ*(*S*_*t*+1_|*θ*^*Q*^) represents the output of the actor-network. As the algorithm also uses a CNN (Convolutional Neural Network) or fully-connected network to approximate the strategy function, it is also called a strategy network whose input is current state *s* and output is action *a*. Nevertheless, the parameters of the policy network are updated to increase the output of the value function network:

$$\max J=\max E_{s-p^{\mu }}[Q(s,\mu_{\theta }(s))]$$ (4)

However, (4) is complicated in practice, and its gradient can be approximately transformed into:

$$\Delta_{\theta \mu }J\approx \frac{1}{N}\sum_{i}\Delta \alpha Q(s,a,|\theta^{Q})|s=s_{i},a=\mu (s_{i})\Delta_{\theta \mu }\mu (s,a|\theta^{\mu })|s_{i}$$ (5)

**Fig 3:** DDPG algorithm based on deep reinforcement leaning.

### 2.4 Target tracking based on CNN

CNN is a feed-forward neural network. The convolution layer’s feature map can track targets. Different layers’ feature maps function differently [19]. Therefore, in target-tracking neural networks, the candidate images should be as few as possible for end-to-end output. The network structure is not simplified to speed up the calculation by the feature vector extracted from CNN. CNN updates each neuronal information, and the feature extraction can be expressed *S*(*x*_*i*_,*w*,*b*). The loss function’s cross-entropy for the *i-*th sample (*x*_*i*_,y_i_) is defined as:

$$L_{i}=‐\ln e^{s_{y_{i}}}+\ln\sum e^{s_{i}}$$ (6)

After a single sample (*x*_*i*_,y_i_) passes through the network, the output should be *f*(*x*). Then, the corresponding loss value should be:

$$L_{i}(f(x),y)=‐\ln f{\left(x\right)}_{y}$$ (7)

CNN’s backpropagation rule updates each neuron’s weight, making the model’s overall error function decrease continuously. The convolution process is defined as follows:

$$x_{j}^{l}=f(\sum_{i\in M_{j}}x_{i}^{l-1}\times k_{ij}^{l}+b_{j}^{l})$$ (8)

In (8), *l* is the convolution layers in the model, $k_{ij}^{l}$ represents the convolution kernel number, $b_{j}^{l}$ is the additive bias, *f* is the activation function, and *M*_*j*_ is the input image. The convolution collection layer can be defined as:

$$x_{j}^{l}=f(\beta_{j}^{l}down(x_{i}^{l-1})+b_{j}^{l})$$ (9)

In (9), *down*(⋅) denotes the data collection function, $\beta_{j}^{l}$ and $b_{j}^{l}$ represent product bias and additive bias, and *f* is the activation function. Its structure is shown in Fig 4.

**Fig 4:** Structure diagram of convolution neural target tracking in table tennis.

### 2.5 Trajectory prediction based on LSTM network

LSTM, a special neural network structure, can process time-series data by recording and processing the first N frames’ inputs and the network’s intermediate results. Thus, it can integrate multiple frames’ information for classification, regression, and input prediction [20]. LSTM’s form is primarily the same as others, consisting of the input layer, hidden layer, and output layer. A hidden layer can contain multiple LSTM units, a unique design form of a hidden layer node of RNN [21]. The detailed internal structure of the unit is shown in Fig 5. The equation of each unit is as follows:

$$f_{t}=\sigma (W_{f}\cdot \left[h_{t-1},x_{t}\right]+b_{f}$$ (10)

In (10), *f*_*t*_ and *i*_*t*_ denote the step *t* forgetting gate and input gate, respectively. In each playing process, the forgetting gate controls each movement process, and the input gate controls each trajectory prediction process.

$$i_{t}=\sigma (W_{i}\cdot \left[h_{t-1},x_{t}\right]+b_{i}$$ (11)

$$C=\tanh(W_{c}\cdot \left[h_{t-1},x_{t}\right]+b_{c}$$ (12)

$$C_{t}=f_{t}\times C_{t-1}+i_{t}\times C$$ (13)

The Sigmoid function is selected for *f*_*t*_ and *i*_*t*_, and the value range is [0,1]. The Tanh function’s value is [–1,1]. *C*_*t*−1_ is the neuron’s state at time *t-1*, and *C*_t_ is the neuron’s state at time *t*.

$$h_{t}=o_{t}\times \tanh(C_{t})$$ (14)

$$o_{t}=\sigma (w_{o}\cdot \left[h_{t-1},x_{t}\right]+b_{o}$$ (15)

In (14) and (15), *o*_*t*_ is the degree that the output gate controls the trajectory, *h*_*t*_ is the output of step *t* in the trajectory.

**Fig 5:** Structure of LSTM unit.

An RNN (Recurrent Neural Network) with LSTM units is built, which receives table tennis ball’s 3D spatial position at time *t* as the input and output at time *t+l*. The input layer receives the ball’s 3D spatial position at time *t* and transmits it to the *n-*th LSTM unit in the hidden layer. Each LSTM unit calculates the current time according to the input and internal state values and outputs the calculation result to the fully-connected layer. Simultaneously, the internal state value is updated and retained until time *t+l*. The specific structure is shown in Fig 6.

**Fig 6:** Structure of table tennis trajectory prediction.

### 2.6 Data training and model evaluation

(1) Experimental environment: the CPU (Central Processing Unit) model is Intel Core i7-4790k. The GPU (Graphics Processing Unit) model is GeForce GTX 1060, with 6GB video memory and 16GB DDR3 memory. The experimental OS (operating system) is Ubuntu 16.04. Pytorch framework implements and debugs the algorithm and compares the differences among different algorithms. Pytorch is an open-source Python machine learning library. Pytorch supports tensor calculation on GPU and can easily write deep learning networks in object-oriented programming. The compiled network supports an automatic differential system for backpropagation and network weight updating. Besides, the visualization tools provided by Tensorflow make the training, debugging, and visualization of DNN (deep neural network) convenient [22].

(2) Data sources: the first is network datasets. Any target detection or tracking algorithm requires marked images or video data to train DNNs or evaluate algorithm performance. Therefore, preparing data is the basis of the algorithm. YouTube-8M is a sizeable marked video dataset containing millions of YouTube videos. It includes thousands of videos under the “table tennis” tag, whose length ranges from 2 to 5 minutes [23]. Second, videos are shot for this experiment. Two static cameras with different view angles are used. The hardware trigger is also specially designed for this experiment, ensuring synchronization. The frame rate includes 50FPS, 100FPS, and 150FPS. In these videos, the background is covered with a white cloth, and table tennis balls are served at a constant speed by a ball machine. The shot videos’ length is about 3s.

Self-built dataset: multiple sets of data under different experimental conditions are taken on the spot, all of which are taken with two stationary cameras with different angles of view, and a self-made hardware trigger is used to ensure synchronization. The shooting frame rate is divided into 50FPS, 100FPS, and 150FPS. The video includes both table tennis using a ball machine to serve at a constant speed, as well as multiple back and forth parts of two people practicing table tennis. Among them, the length of the video using the ball machine is about 3s, and the background is a black cloth to distinguish it from the white table tennis ball, which is less difficult. In the video of two people practicing table tennis, the background is not treated or processed. However, there is no additional object change in the background, which is slightly more difficult. The data source of the training target detection algorithm is divided into two parts. There are unlabeled table tennis images in ImageNet, which are downloaded and labeled using the written auxiliary program. In addition, from the directly shot videos, the position of the table tennis ball in each frame of the image is marked first. Then the generated images are randomly cropped and added with noise to generate more data. Some of these data include table tennis balls while some do not, all of which are utilized for training the target detection algorithm. Finally, about 4,000 positive sample images and 4,000 negative sample images are produced. The specific scenarios are shown in Fig 7.

**Fig 7:** Real-time data acquisition system.

(3) Model training: the detection algorithm has two data sources. ImageNet contains unmarked images. After these images are downloaded, an auxiliary program is launched to mark them. The ball’s position in each frame is marked from the video taken directly. Afterward, the images are randomly cropped, which are then added with noise to generate more data. Some data include the ball’s information, while some do not, which are adopted to train the detection algorithm. Finally, about 4,000 positive and 4,000 negative image samples are generated. The training and testing data are at the ratio of 8:2.

(4) Performance evaluation: when the ball hits the table, the central mass’ height *z* is equal to the ball’s radius. At this moment, only the *x* and *y* dimensions are considered to reduce the hitting point’s error. The prediction results at the hitting point can reflect the prediction method’s accuracy and adaptability. MSE (Mean Squared Error) and RMSE (Root Mean Squared Error) evaluate the same dataset [24]. ACC (Accuracy), Pre (Precision), and F-measure are criteria for evaluating model performance [25]. SD (Standard Deviation) is the variance between the predicted value and the mean predicted value.

$$MSE=\frac{1}{N}\sum_{i=1}^{N}(A_{i}‐B_{i}{)}^{2}$$ (16)

$$RMSE=\sqrt{\frac{1}{N}\sum_{i=1}^{N}(A_{i}‐B_{i}{)}^{2}}$$ (17)

In (16) and (17), *A*_*i*_ represents the original dataset, *B*_*i*_ represents the prediction dataset, *A* represents the mean predicted value, *ACC* represents the recognizable trajectories’ proportion in the total recognition, *Pre* represents the positive categories’ proportion in the recognized samples, F-measure represents the weighted harmonic mean of the accuracy rate and recall rate, which evaluates the quality of the classification model, and *Rec* is the model’s recall rate:

$$ACC=\frac{TP+TN}{TP+FP+FN+TN}$$ (18)

$$\mathrm{Pr}ecision=\frac{TP}{FP+TP}$$ (19)

F‐measure=2*Pre*RecPre+Rec (20)

In (18) and (19), *TP* represents the number of correlated positive categories retrieved. FP represents the number of uncorrelated negative categories retrieved. *FN* represents the number of uncorrelated positive categories not retrieved, and *TN* represents the number of uncorrelated negative categories not retrieved. MSE and RMSE show the prediction accuracy. The smaller the MSE and RMSE, the higher the prediction accuracy. SD suggests the predicted value’s dispersion degree. The smaller the SD, the more concentrated the predicted value, the smaller the probability of a large deviation of the predicted value from the actual value, and the better the prediction method’s adaptability.

## 3. Results

### 3.1 Feature extraction results based on deep reinforcement leaning

Fig 8 shows a comparison of different feature extraction algorithms. The performance differences of different algorithms are quite different in accuracy, precision, and comprehensive evaluation performance. DDPG algorithm has the best performance among feature extraction algorithms, and the maximum accuracy rate can reach 89%. The same error results also show that the DDPG algorithm is more accurate than others, and its minimum MSE is 0.2475. Therefore, the proposed deep reinforcement leaning can accurately extract features and significantly improve the model’s performance.

**Fig 8:** Feature extraction results based on deep reinforcement leaning. Note: common feature extraction algorithms include SIFT (Scale Invariant Feature), SURF (Speeded Up Robust Feature), ORB (ORiented Brief), FAST, and DPG (Deterministic Policy Gradient).

### 3.2 Target tracking results based on CNN

Fig 9 suggests that as iteration continues, the models’ performance is improved continuously. All the algorithms are compared. The algorithm model using a neural network is better than the traditional method using probability. CNN target tracking algorithm has the highest performance, and the accuracy is 93%. Error results also show that the CNN target tracking algorithm is more accurate than other algorithms. Hence, the proposed model’s target tracking results are fair.

**Fig 9:** Target tracking results based on CNN. Note: common target tracking algorithms include CF (Collaborative Filtering), DPN (Deformable Parts Model), SVM (Support Vector Machine), RPN (RPN+Fast RCNN), and YOLO (You Only Look Once).

### 3.3 Trajectory prediction results based on LSTM network

Fig 10 shows that as iteration continues, the models’ performance is improved continuously. All the trajectory prediction algorithms are compared. LSTM is superior to other algorithms. The maximum accuracy can reach 91%, and the minimum error is 0.5117. The above results show that the proposed trajectory prediction model based on the LSTM network is useful and has made significant improvements in table tennis’s trajectory prediction.

**Fig 10:** Trajectory prediction results based on LSTM network. Note: common trajectory prediction algorithms include ID3 (Iterative Dichotomiser 3), BP (Backpropagation), RNN, ARIMA (Autoregressive Integrated Moving Average model), and Kalman gain.

### 3.4 Overall performance evaluation of the model

Fig 11 shows the comparison results between the fusion model and the traditional method. Compared with the traditional method, the precision and accuracy of the DCNN-LSTM (Deep Convolutional Neural Network Long Short Term Memory) model based on deep learning is improved by 23.17% and 14.57%, respectively. The MSE and the average MSE decreases by 65.13% and 7.19%, respectively. The above results show that the proposed tactical indicator automatic detection model’s performance is significantly improved than the traditional methods.

**Fig 11:** Overall performance evaluation results of the model. Note: TM represents the traditional detection method of table tennis tactical indicators, and DCNN-LSTM represents the fusion algorithm model in DDPG+CNN+LSTM.

## 4. Conclusion

The proposed real-time detection algorithm based on deep learning can eliminate the target background, extract the target features, and track and detect table tennis balls, presenting excellent real-time performance. The LSTM network and multiple models are fused, which significantly improves the prediction accuracy. Finally, a model system is built for predicting the ball’s spatial position, which solves the problems in the traditional prediction view-points. The proposed deep learning-based algorithm effectively settles the difficulties in existing table tennis’s tactical estimation, providing new ideas for the tactics research. Nevertheless, some deficiencies are found: first, the proposed algorithm is only effective in simulation experiments. Because the theoretical model may have some practical application errors, the model’s parameters need to be optimized continuously. Second, the proposed algorithm is proved to be effective. However, this will have higher requirements for the migration ability and operating environment of the system. Therefore, the fusion model’s fitness needs improving, and the system’s energy consumption needs reducing. In the future, the above two aspects will be analyzed profoundly further to improve the system’s detection performance for ball games.

## Supporting information

S1 Data (RAR)
